# Influence of Taijiquan Exercise on Mentality and Emotion Regulation by Intelligent Medical Big Data Analysis

**DOI:** 10.1155/2022/5468317

**Published:** 2022-10-11

**Authors:** Shuaiju Han, Shaohui Hu, Kang Li

**Affiliations:** ^1^Department of Physical Education, Graduate School, Sejong University, Seoul 04989, Republic of Korea; ^2^Beijing Sport University China Wushu School, Beijing 100084, China; ^3^Physical Education Department, Tianjin Vocational and Technical Normal University, Tianjin 300222, China

## Abstract

Taijiquan training emphasizes the relaxation of the mind and the body, pay attention to maintain the peace of mind, and minimize the impact of external interference on the body so as to make the mind more comfortable. This study mainly explores the influence of Taijiquan practice on emotion regulation based on intelligent medical health big data analysis. The significance of Taijiquan in developing and improving the positive emotions of middle-aged people and maintaining physical and mental health is expounded. There are two methods of data collection: full collection and incremental collection. In this study, when the psychological testing equipment was launched, a full amount of historical data was collected; after the psychological testing equipment was online, the collection method was generally carried out in the way of incremental collection. The subjects exercised Taijiquan three times a week, one hour each time, and the exercise content was the 24-style Taijiquan designated by the workstation. At the same time, the subjects were asked not to engage in other regular physical exercise projects in their spare time. By longitudinal tracking and comparison of the Taijiquan intervention group after participating in the Taijiquan exercise intervention, the differences in the state of mind and emotion regulation strategies, and 12 subjects were selected voluntarily to participate in the emotional Stroop (the color words used in the classic Stroop paradigm were replaced with emotional and nonemotional words written in different colors, and the subjects were still tasked with responding to colors) experimental paradigm. In this paper, the moderate-intensity Taijiquan project is selected, which is in line with the effective value threshold theory of exercise load. It studies the effects of exercise on the body shape, cardiopulmonary function, flexibility, and balance ability of the body according to the metabolism theory and the movement balance theory of the human body adapting to the environment. Before the experiment, there was no significant difference between the Taijiquan training group and the control group, but after the experiment, there was a significant difference between the Taijiquan training group and the control group (*P*<0.05). Taijiquan has a significant effect on improving students' body shape, cardiopulmonary function, flexibility, balance, and mood.

## 1. Introduction

In the development of national sports, the research on sports and psychology has become a research hotspot nowadays, while the impact of Taijiquan on people's mental health in the related research on Taijiquan is still relatively limited. The empirical research needs more scientific and rigorous theoretical support. With the deepening of people's understanding of mental health, the factor of “emotion” has a stronger practical value and positive significance in improving human health. Positive emotion is an important part of the research field of positive psychology, and it plays an extremely important role in promoting the development of people's mental health. Those who practice Tai Chi regularly can coordinate and unify the functional activities of various organs in the whole body and enhance the body's ability to adapt to environmental changes. Through the strengthening of myocardial contractility and the increase of blood output, Tai Chi exercise can also improve the utilization rate of oxygen in various organs and tissues in the body, improve the exchange efficiency of substances inside and outside the capillaries, and promote the metabolism of substances in the body. Taijiquan emphasizes the characteristics of circular arcs in the route and posture and the characteristics of body movement so as to achieve coherence and twists and turns. In the whole training process, each part of the body has different degrees of circular movements in harmony, so that the muscles, ligaments, and bones of the whole body can be properly and evenly exercised. Positive emotions prompt human beings to produce more new positive thoughts and positive behaviors in social practice, which is consistent with the pursuit of comprehensive and healthy development in today's era. Therefore, it is a good way and method to use sports as a carrier to help people experience more positive emotions and develop people's enthusiasm, creativity, and innovation. Combining Taijiquan with emotions in the field of psychology will enrich the theoretical research on the effects of Taijiquan on people's mental health in Taijiquan. Therefore, it is quite necessary to conduct research on the influence of Taijiquan on the positive emotions of middle-aged people. Tai Chi is a safe, feasible, and effective form of exercise to improve sleep quality, anxiety, and fatigue.

This paper uses the intelligent medical and health big data technology system to explore the internal mechanism of Taijiquan's influence on people's state of mind and emotional regulation and contributes to the promotion and popularization of Taijiquan; secondly, through the horizontal comparative analysis and longitudinal tracking research, while exploring the characteristics of changes in emotion and emotion regulation strategies, it provides a theoretical basis for the implementation of reasonable physical exercise intervention behaviors; and finally, the research process of this paper is the intervention process of Taijiquan exercise for college students, and the experience data of college students' exercise behavior intervention can be obtained, thereby promoting Chinese traditional sports programs and making college students to participate in physical exercise. It has important practical value in relieving college students' health expenditure pressure and improving college students' physical and mental health and quality of life. During the intervention period, there was a significant difference between the Taijiquan training group and the blank control group (*P* = 0.038 < 0.05).

## 2. Related Work

Taijiquan practice involves left rotation and right rotation, with the waist as the axis, so that the muscles, joints, and even internal organs of the whole body can be properly and evenly moved. At the same time, the gentle, deep, even, and powerful breathing during the training process makes the mind, qi, and force achieve an effective unity, thereby promoting the exhalation of the old and the new, strengthening the circulation of qi and blood in the whole body, and then improving the transportation and transformation efficiency of the subtle substances in the body. Bo et al. believe that data-intensive analytics is a major challenge for smart cities due to the ubiquitous deployment of various sensors. The natural characteristics of geographic distribution require a new computing paradigm to provide location-aware and latency-sensitive monitoring and intelligent control. Fog computing, which extends computing to the edge of the network, meets this need. They introduced a layered distributed fog computing architecture to support the integration of numerous infrastructure components and services in future smart cities. To protect future communities, it is necessary to integrate intelligence into fog computing architectures. For example, it performs data representation and feature extraction, identifies abnormal and hazardous events, and provides optimal response and control. They analyzed case studies using an intelligent pipeline monitoring system based on fiber optic sensors and sequential learning algorithms to detect incidents that threaten pipeline safety. It builds a working prototype to experimentally evaluate event detection performance [1]. Almobaideen et al. believe that tourists with chronic medical conditions are afraid of unexpected emergencies and may be less inclined to travel to remote destinations due to health concerns, especially while on the road. Smartphones, sensor devices, cellular communications, and the Internet of things (IoT) are the latest technologies to deliver new mobile location-based services. Such services can help mobile tourists, those currently moving between locations, access innovative services that make their travel easier and safer. Designing effective solutions to help tourists with chronic illnesses find appropriate geographic routes from source to tourist destination through transportation networks is critical to healthcare systems. They proposed a new method to generate the most suitable geographic routes for proximity to medical centers. Their method, called Geographic Routes for Mobile Tourism (GRMT), selects a route that best suits a medical center and takes the shortest possible path in terms of distance [2]. Lin et al. believe that gait analysis is an important medical diagnostic process with many applications in healthcare, rehabilitation, therapy, and sports training. However, typical gait analysis must be performed in a gait laboratory, which is inaccessible for large populations and does not provide natural gait measurements. They proposed a novel sensor device, the smart insole, to address the challenge of effective gait monitoring in real life. A series of electronic textile (e-textile)-based pressure sensors are integrated into the insole to comprehensively measure plantar pressure. The smart insole is also equipped with a low-cost inertial measurement unit that includes a three-axis accelerometer, a three-axis gyroscope, and a three-axis magnetometer to capture gait characteristics in motion. The smart insole can provide accurate gait information collection. At the same time, it is lightweight, thin, and comfortable to wear, providing an unobtrusive way to perform gait monitoring. In addition, they developed a smartphone GUI developed to display sensor data in real time via Bluetooth Low Energy [3]. Karlowsky et al. believe that Gram-negative ESKAPE pathogens (*Enterococcus faecium*, *Staphylococcus aureus*, *Klebsiella pneumoniae*, *Acinetobacter baumannii*, *Pseudomonas aeruginosa*, and *Enterobacter* species) are responsible for the global increase in drug-resistant infections. They used clinical and laboratory standard research microdilution methods to determine the effect of Gram-negative ESKAPE pathogens isolated from hospitalized patients with intra-abdominal infection (IAI) (*n* = 3052) and urinary tract infection (UTI) on eight parenteral antimicrobials *in vitro* sensitivity [4]. Hou et al. believe that, today, lateral flow immunochromatographic assays are gaining popularity as a diagnostic tool for point-of-care (POC) tests based on their simplicity, specificity, and sensitivity. Therefore, medical testing urgently needs quantitative testing and diversified popularization applications. They developed a smartphone-based dual-modality imaging system for quantitative detection of color or fluorescent lateral flow test strips that can be operated anytime, anywhere. In this system, the optics are designed for white light and ultraviolet (UV) light, which can be tuned through different bands. The Sobel operator algorithm is used in the software to enhance the ability to identify the test area. Furthermore, the technique is based on extracting components from the RGB format of the color bars (red, green, blue) or the red format of the fluorescent bars only, which can significantly improve the signal strength and sensitivity [5]. Taijiquan exercise adopts abdominal breathing, which enhances intestinal peristalsis while exercising, and promotes the transformation of spleen. When practicing boxing, the rhythmic slow, deep breathing can make the lung's function of dispersing, sending, and descending fully exerted, so that the water channel can be adjusted and the lung's defense can be solidified. The public's love for Taijiquan, a mass event that unifies the body and mind and promotes physical health, continues to deepen. This traditional sports event regardless of gender and age is developing rapidly. At the national level, Taijiquan is promoted as a priority.

## 3. Intelligent Medical Health Big Data Analysis Method of Influence of Taijiquan Practice on Emotion

### 3.1. Emotion

All human life activities related to body or spirit are closely related to emotions and have a huge impact. Too strong or persistent negative emotional response will seriously affect the function of the nervous system, especially the damage to the sympathetic and parasympathetic nerves, resulting in an imbalance of neural activity, which leads to the occurrence of various physical and mental diseases. Emotion can reflect a person's emotional state, and the emotional state directly affects people's mental health. Emotions are divided into positive emotion and negative emotion. In a positive state of mind, people can devote themselves to their daily work and life in a relaxed, happy, and full-of-energy manner; communicate actively with others; and strengthen their determination to overcome difficulties, thus contributing to the smooth completion of work; in a negative state of mind, people feel depressed, communicate poorly with others, easily lose confidence, and are often in a state of tension and anxiety, resulting in poor work efficiency [6, 7]. Therefore, the state of mind is closely related to people's mental health. A good state of mind can help to exert initiative and promote mental health, whereas a bad state of mind can easily lead to depression, leading to various mental diseases [8, 9].

Covariance is often used to measure the overall error of two variables in statistical analysis or data mining (the process of searching for information hidden in a large amount of data through algorithms), and the calculation formula is as follows [10]:

(1) $$\begin{array}{c} COV\left(X,Y\right)=\sum^{}\left(X-\right)\left(Y-\right). \end{array}$$

And according to the different values of covariance, it has the following conclusions [11]:

(2) $$\begin{array}{c} COV\left(X,Y\right)=\left\{\begin{array}{c} >0,X,Y\text{ positive correlation},\\ <0,X,Y\text{ negative correlation},\\ =0,X,Y\text{ are independent of each other}. \end{array}\right. \end{array}$$

The correlation coefficient *R* needs to be used to measure and compare the closeness of the correlation [12]:

(3) $$\begin{array}{c} R=\frac{S_{XY}}{S_{X}S_{Y}}, \end{array}$$

where *S*_*X*_ and *S*_*Y*_ represent the sample standard deviations of *X* and *Y*, respectively.

The min-max normalization formula is used [13]:

(4) $$\begin{array}{c} v=\frac{v-{\text{min}}_{a}}{{\text{max}}_{a}-{\text{min}}_{a}}\left(\text{new}\_{\text{max}}_{a}-\text{new}\_{\text{min}}_{a}\right)+{\text{min}}_{a}. \end{array}$$

The range of attribute *a* can be converted to interval [new_min_*a*_, new_max_*a*_].

Z-score normalization [14]:

(5) $$\begin{array}{c} v=\frac{\left(-a\right)}{\beta_{a}}, \end{array}$$

where $\bar{v}$ is the mean of *v*.

Classification accuracy calculation formula [15]:

(6) $$\begin{array}{c} \text{accuracy}=\frac{\left(TP+TN\right)}{\left(P+N\right)}. \end{array}$$

The horizontal and vertical coordinates are FPR and TPR [16]:

(7) $$\begin{array}{c} \text{FPR}=\frac{FP}{\left(FP+TN\right)},\\ \text{TPR}=\frac{TP}{\left(TP+TN\right)}. \end{array}$$

The calculation method of *F*1-Measure is as follows [17]:

(8) $$\begin{array}{c} P_{R}=\frac{TP}{\left(TP+FP\right)},\\ R_{E}=\frac{TP}{\left(TP+FN\right)},\\ F_{1}=\frac{2{}^{*}R_{E}{}^{*}P_{R}}{\left(R_{E}+P_{R}\right)}. \end{array}$$

For the classification results, *P*_*R*_ and *R*_*E*_ are of course the higher the better.

The formula for constructing a new sample is as follows [18]:

(9) $$\begin{array}{c} p_{ij}=x_{i}+r\left(0,1\right)*\left(y_{ij}-x_{i}\right), \end{array}$$

where *x*_*i*_ represents a minority class sample.

### 3.2. Selection of Experimental Subjects

The physical and psychological conditions of college students are basically in the late stage of development, and various physiological and psychological indicators are gradually stable and mature [19, 20]. This experiment requires the participants to be healthy, develop normally, have no contraindications to exercise, have a good living condition, have no history of systematic exercise, have no history of disease, and have not performed simplified Taijiquan-related exercises in the past. The subjects were divided into the experimental group of 40 and the control group of 40 (both were 20 males and 20 females). During the whole experiment period, the experimental subjects should obey the experimental plan and understand the content and purpose of the experiment. Among them, the students in the experimental group participated in the experimental control. In order to ensure the scientificity of the experiment, only simplified Taijiquan exercise intervention was conducted during the experimental period and no other sports were allowed. The students in the control group did not engage in any physical activity except for daily study. The subjects maintained a normal diet during the experimental period.

### 3.3. Embodiment of Regular Practice

The so-called regular Taijiquan practice is a scientific and reasonable arrangement of Taijiquan practice time, practice frequency, exercise load, etc. In this experiment, Panorama Campus was selected as the research site. If only experimental research is carried out in the physical education class (3 sessions per class per week), it is difficult to reflect the regularity in the time, frequency, and load of practice. Due to the specific circumstances of the school's sports activities, in addition to physical education classes, there will be 28-minute group interclass activities in the morning and afternoon every day (mainly in class laps and rope skipping). Through the application with the school's physical education teachers and school leaders, it was finally determined that the third and fourth grade classes would be the experimental research objects. This experiment mainly uses the exercise time between classes to carry out the experiment and conducts a certain degree of guidance in the physical education class without affecting the normal physical education curriculum.

The experimental practice period is from Monday to Friday, for a period of 14 weeks. It mainly uses the morning and afternoon exercise time to intervene, to ensure that the daily practice time is not less than 25 min, and the exercise intensity and load are subject to subjective adjustment according to the specific mastery of students' learning. The progress of Tai Chi teaching is shown in Table 1.

### 3.4. Literature Search

According to the research purpose and research content, through literature retrieval (the process of obtaining literature according to the needs of study and work), network retrieval, etc., read a large number of papers on concept definition and emotional characteristics of college students, emotion and emotional regulation theory, Taijiquan exercise theory and its effect on physical and mental effects, physical exercise statistics, etc. and writings. And this paper collects domestic and foreign literature related to this subject, grasps the research situation at home and abroad, and provides a theoretical basis for the research of this paper.

### 3.5. Psychometrics

#### 3.5.1. Measuring Tool

According to the research content, following the requirements of sports scientific research methods and questionnaire design, the “Questionnaire on the Effects of Taijiquan Exercise on Emotion and Emotion Regulation” was designed. The questionnaire includes the following: the first part is the basic information, including the district/county, gender, age, current living situation, reason for participating in physical exercise, years of Tai Chi exercise, number of weekly exercises, time of each exercise, etc.; the second part is the brief mood scale (POMS); and the third part is the Emotion Regulation Questionnaire (ERQ).

#### 3.5.2. Psychometric Procedures

With the help of the school's martial arts teachers, contact and negotiate with the heads of each Taijiquan workstation and organize the distribution of questionnaires on the spot after the morning practice of college students. First of all, it explains to the respondents the purpose of the survey, the purpose and significance of this research, and the commitment to confidentiality of personal information, so as to improve the cooperation of the respondents and the authenticity of the questionnaire. Then, the way to fill in the questionnaire is carefully described, and the survey assistant will explain in time the questions that the college students cannot understand. The person in charge will read out the questions one by one and fill in them after asking and verifying. After completing the questionnaire, the on-site recovery was carried out to improve the standardization and accuracy of the questionnaire filling. In the process of questionnaire recovery, the researchers explained and corrected the respondents in a timely manner for the incomplete and missing items in the questionnaire to ensure the integrity of the survey data and gave small gifts after the effective questionnaire was recovered.

### 3.6. Experimental Study

#### 3.6.1. Experimental Equipment

This experiment was carried out in the Psychological Experiment Evaluation Room of the Department of Health Sciences, which sound insulation, ventilation, temperature, and humidity are good. The computer screen is 44 cm long and 30 cm wide, the screen resolution is 1280 × 760, the true color is 32 bits, and the screen refresh rate is 60 Hz.

#### 3.6.2. Experimental Design and Principle

This experiment adopts the classical emotion Stroop paradigm. The design of this experiment is a single-factor between-subjects design. The factor is the magnetism of priming vocabulary, including positive vocabulary, neutral vocabulary, and negative vocabulary. The dependent variables are the response time and the correct rate. The overall architecture of the medical big data analysis and intelligent supervision system can be divided into four main parts: scheduling service (referred to as scheduling or ETL), analysis and supervision rule engine (referred to as engine), business data warehouse, and application services. The logical structure of medical big data is shown in Figure 1.

#### 3.6.3. Vocabulary Filter

1. 136 emotional words and nonemotional words with no significant difference in word frequency were selected according to the “Modern Chinese Common Words Dictionary” and “Modern Chinese Commonly Used Words Word Frequency Dictionary”.
2. The 136 words were evaluated by 5 Chinese language teachers and 20 middle school students on the nature of words (positive-neutral-negative). After the evaluation test, 60 candidate words were selected according to the frequency of word occurrence.
3. Finally, they were filtered through vocabulary familiarity (familiar-common-rare) and parts of speech (adjective or noun).

#### 3.6.4. Experimental Operation

With the help of the community staff and the organizers of the Taijiquan activity station, after the screening of the questionnaire, this paper selects the “24-style Taijiquan” commonly used in the activity station as the exercise method for the intervention experiment. It requires at least 60 minutes of exercise at least 3 times a week for 6 months. During this period, the subjects were required not to participate in other regular exercise, and they had to perform planned Taijiquan exercise according to the prescribed exercise frequency, intensity, and time each week. In case of special circumstances, such as illness, weather, and other uncontrollable factors, the exercise plan can be adjusted appropriately. An experimental test is conducted every two months; the first test is on September 12, 2017, the second test is on November 14, 2017, and the third test is on January 10, 2018. The records were extracted and saved three times for statistical analysis, and a small gift was distributed to the subjects at the end of each test.

#### 3.6.5. Experimental Procedure

This experiment was written by E-Prime software, and the computer automatically recorded the response time and accuracy of the subjects. The experiments were carried out in a light-controlled semi-soundproof laboratory. The subjects sat on a chair, facing the computer screen, with their eyes about 60 cm away from the screen, and the subjects were required to keep their eyes on the center of the screen during the experiment. Before the experiment, the subjects were said to relax during the experiment, not to guess the experimenter's purpose, just follow the experimental instructions; when it is ready, press the “Space” key to perform the practice test and then start the formal experiment.

#### 3.6.6. Data Acquisition Link

The extraction link of data acquisition is to use the data acquisition interface to connect the ETL and the database of the hospital information system for communication. A variety of interactive methods can be adopted for the specific implementation. The interaction frequency has been analyzed in the previous article, and the incremental extraction method can be adopted once a day (or weekly). ETL extracts the data through the data acquisition interface, cleans the data as needed, normalizes the nonstandard data, and removes the impurity data. It writes the cleaned data to the MongoDB (a database based on distributed file storage) database server. The network topology is shown in Figure 2.

As can be seen from Figure 2, the system includes two large functional modules, namely the acquisition part of the machine learning model and the decision support part. The machine learning model acquisition part is used to train mathematical models for different diseases, and the obtained models are stored in the database in the form of mathematical parameters, and doctors can study and train the required models in their spare time. In the actual diagnosis and treatment process, what doctors use is the decision support (assist decision-makers in semistructured or unstructured decision-making in a human-computer interaction manner through data, models, and knowledge) part, and the system reads the actual clinical data of the patient and brings it into the relevant trained model for calculation, so as to obtain the necessary decision-making suggestions. This suggestion may be a diagnosis suggestion of a disease, a suggestion of an examination item to be performed, a suggestion of a prescription drug treatment, a suggestion of an anesthesia dose, and so on. These suggestions depend on the models in the system, which means that the more models that doctors train, the more suggestions they can get from the system. After getting the advice, the doctor can also give feedback to the suggestion given by the system according to the design situation observed by him, and the system will automatically train and update the model parameters online based on the feedback and the new related data collected recently. This clinical decision support system does not contain any knowledge at first, only the machine learning algorithm framework. However, with the continuous use of the system, a large number of models with different functions will be trained and the models will be continuously updated according to the actual situation. It can be said that the system will gradually accumulate a large amount of knowledge, and the knowledge will be updated dynamically with the change of the actual situation, and the knowledge contained in the system is constantly growing and changing.

The transfer function is given in the following formula [21]:

(10) $$\begin{array}{c} S_{D}=\sum^{}P_{i},\\ S_{ni}=\sum^{}y_{i}P_{i}. \end{array}$$

The number of neurons in the output layer is the dimension of the output vector in the learning sample, and the *j*th neuron corresponds to the *j*th element of the prediction result. The calculation method is as follows [22]:

(11) $$\begin{array}{c} y_{i}=\frac{S_{ni}}{S_{D}}. \end{array}$$

One neuron in the pattern layer corresponds to one learning sample [23]:

(12) $$\begin{array}{c} p_{i}=\exp\left[-\frac{{\left(x_{i}-x_{n}\right)}^{T}\left(x_{i}+x_{n}\right)}{2\sigma^{2}}\right]. \end{array}$$

This parallel processing method *ERR* can improve the computational efficiency several times [24].

(13) $$\begin{array}{c} ERR=\overset{N}{\underset{i=1}{\sum }}w_{i}\left[y_{i}\neq g\left(x_{i}\right)\right]. \end{array}$$

The classification result of the new sample is the weighted sum *G*(*X*) of the classification results of *T* decision stump submodels [25]:

(14) $$\begin{array}{c} \alpha =\log\sqrt{\frac{\left(1-\varepsilon \right)}{\varepsilon }},G\left(X\right)=\text{sig}\left(\sum^{}\alpha_{t}\times g_{t}\left(X\right)\right), \end{array}$$

where *α* is the weighting factor. Finally, the *C* values are copied back to the CPU to complete the final accumulation operation, and the final target value *J* is obtained.

(15) $$\begin{array}{c} J=\overset{C}{\underset{i=1}{\sum }}\overset{N}{\underset{K=1}{\sum }}{\left(UK\right)}_{M}{\left(D_{i,k}\right)}^{2}. \end{array}$$

The whole experiment time is about 15 minutes. In the formal experimental stage, the process of each trial is as follows: first, a black “+” fixation point (font Courier New, font size 48) will appear in the center of the computer screen to help the subject concentrate, and it will disappear after the presentation time is 1000 ms; then the vocabulary (font italic, font size 48) appears in the center of the screen, and the presentation time is unlimited, that is, the subject responds to the color of the vocabulary and responds to the button, and the stimulus disappears; next a white blank screen is presented as a buffer, the presentation time is 500 ms, and then it is the next trial [26].

*ERP data* was recorded by Brain Product's Brain Vision Recorder software and then analyzed using Brain Vision Analyzer [27].

### 3.7. Mathematical Statistics

The statistical software Spss17.0 was used to perform descriptive statistics, one-way analysis of variance (ANOVA) and paired samples t-test were used on the collected scores of the POMS Scale of Mood and the Emotion Regulation Questionnaire (ERQ), as well as the three data measured before and after the E-Prime experimental intervention were analyzed using one-way ANOVA and paired samples t-test.

## 4. The Effect of Taijiquan Practice on the State of Mind

During the intervention period, there was a significant difference between the Taijiquan training group and the blank control group (*Z* = −2.070, *P* = 0.038 < 0.05). The comparison of different intervention time between Taijiquan training group and blank control group is shown in Table 2.

The GSES (General Self-Efficacy Scale–Schwarzer) score was tested using the *t*-test, and there was no significant difference between the Taijiquan training group and the blank control group (*t* = −1.065, *P* = 0.288 > 0.05). The GSES score results are shown in Table 3.

The comparison of SCL90 score results is shown in Table 4.

The change value of the height and weight of males and females in the third-grade experimental class was *P*<0.05, indicating that the height and weight of the male and female students in the experimental class increased to varying degrees compared with those before the experiment. Especially in the experimental class, *P*<0.01 in height, indicating a very significant difference; the change value of the height and weight index of girls in the control class was *P*<0.05, indicating that the two indexes of girls before and after the experiment changed significantly. The height change of the boys in the control class was *P*<0.05, the difference was significant, and the weight change was *P*<0.05, indicating that the weight of the boys in the control class changed significantly. Before and after the third-grade experiment, the comparison of the height and weight indicators of the experimental class and the control class is shown in Figure 3.

The average change of height and weight of fourth-grade students is shown in Figure 4. The height of the boys in the experimental class increased by 1.02 cm, whereas the height of the boys in the control class increased by 0.73 cm, and the increase in the experimental class was 0.29 more than that in the control class; the weight of the boys in the experimental class increased by 0.4 kg, while that of the boys in the control class increased by 0.51 kg, and the increase in the experimental class was greater than that in the control class. The height of the girls in the experimental class increased by 2.275 cm, whereas the height of the girls in the control class increased by 1.69 cm, and the increase in the experimental class was greater than that in the control class; the weight of the girls in the experimental class increased by 0.92 kg, while that in the control class was 0.714 kg, and the increase in the experimental class was 0.179 kg more than that in the control class.

The height and weight indexes of the third- and fourth-grade students before the experiment were compared with each other, and the results showed that the Sig (two-sided, it may be greater than and may be less than) values were all greater than 0.05 (*P*>0.05). Before the experiment, the height and weight of the students in the experimental class and the control class were compared with each other, as shown in Table 5.

The intervention program significantly improved the 50 m running of the third- and fourth-grade students (*P*<0.05), indicating that regular physical activity has a certain effect on the improvement of the speed quality of the students in this grade. The comparison of the 50 m running time between the third- and the fourth-grade students is shown in Figure 5.

The comparison between the third-grade experimental class and the control class showed that *P*<0.05, with a significant difference, but the experimental class *P*<0.01, and the difference was very significant. Comparing the changes of the mean value of the experimental class and the control class, it can be seen that the mean value of the experimental class has a larger increase than that of the control class; there was no significant difference between the groups before the experiment, and there was a significant difference between the groups after the experiment (*P*<0.05). Therefore, we can conclude that Taijiquan has a significant effect on increasing the stamina of third-grade students. The results of the students' physical fitness test are shown in Figure 6.

By posting posters in the school, as well as the recommendation of teachers and parents, the tests of the early emotional intelligence scale (which is an indicator of a person's mood, level, or state of emotional development) and emotion self-rating scale of the applicants were conducted, and the total emotional intelligence score from low to high and the emotion self-rating total score were ranked and sorted from high to low (the lower the emotional intelligence total score, the higher the emotion self-rating total score, indicating more negative emotions, weaker ability to regulate and control emotions, and poorer emotional state). 12 students with poor emotional state in the front row were screened out as the participants of this emotional improvement group. Among these 12 people, the total score of emotion self-assessment was significantly higher than that of other peer groups, and the total score of emotional intelligence was significantly lower than that of other peer groups. Therefore, the group participants have more negative emotions and poorer state of mind and need timely intervention. They try to help clients find and analyze the stressors that cause negative emotional reactions through the development of emotion improvement groups, improve their ability to solve and deal with problems, and affirm their strengths and progress, so as to improve their emotional state. The state of mind of the 12 people is shown in Figure 7.

The group members were tested before and after using the emotional intelligence scale to examine the intervention effect of group work on the level of emotional intelligence. The statistical results are shown in Figure 8. A good grasp of emotional perception in emotional intelligence can be seen after the test.

Compared with the control group, there were significant differences in the factors of activity, depression, and inactivity between the Taijiquan experimental group and the control group. The comparison of emotion factors is shown in Table 6.

The emotion self-rating scale was used to investigate the changes of emotion of the members before and after the activity. The emotion self-rating scale is divided into two parts: positive emotion and negative emotion.  Figure 9 shows the effect of group work on the improvement of group members' emotion and the statistical results of each dimension of the self-assessment of emotion.

The negative emotions of the group members, such as nervousness, anger, fatigue, depression, and panic, decreased significantly after the activity, while the scores of positive emotions of energy and self-esteem increased significantly. The total score of emotion decreased significantly, indicating that this group work is not only an effective method for self-adjustment of emotion but also an important method to successfully improve vitality and reduce tension. In the group, the team members confided their worries, sorrows, anger, and other feelings and obtained the empathy, support, and help of other team members and social workers, thus enriching the personal support network, allowing the team members to relieve pressure, improve self-confidence, and enhance resilience. “Emotional catharsis and regulation” allows team members to learn to deal with and control their own emotions independently and apply them to their own lives to reduce negative emotions. Through the eight-style Taijiquan learning, the team members can relax physically and mentally from these slow, stretching, and smooth movements. The visual movements combined with quiet breathing can vent and sublimate negative emotions. At the same time, in the process of exercising, we constantly learn new movements and create new opportunities for challenges. Through the help of teachers and team members as well as personal efforts, success and affirmation in challenges is an important way for team members to build self-confidence. Therefore, the positive emotions of the group members were improved, and the emotion state was improved.

## 5. Discussion

As a treasure of traditional Chinese culture, Taijiquan is known as the physical expression of traditional Chinese philosophy and the best fitness exercise in the world. Due to the research on the medical effect of Taijiquan in recent years, the curative effect of Taijiquan has been paid more and more attention by the international medical community. Taijiquan practice pays attention to relaxation, tranquility, and stability, leading the qi with the mind, and the strength is sent from the abdomen to the limbs, which promotes automatic massage inside the body and promotes metabolism. Regular Tai Chi practice can maintain the toughness of skeletal muscles and promote the nutritional status of tissues around joints. People who persist in practicing Taijiquan for a long time not only have a healthy body but also have a positive mental state. It can be seen that Taijiquan has a good effect on improving physical fitness.

Taijiquan takes the waist as the axis, emphasizing the role of the waist in the way of boxing, and a large number of arc-shaped spiral movements play a role in massaging the waist and abdomen. There is a folk proverb saying that if you do not revitalize your waist, you will not be skilled in the end, emphasizing the importance of the waist in martial arts practice, and Taijiquan is an effective means to develop the waist movement of humans. Taijiquan pays attention to the external relaxation and internal tightness, and the external posture is relaxed. In fact, many muscles in the body are in a state of contraction and exertion, which has higher requirements for muscle contraction and relaxation functions, and movements such as body rotation, independence, and kicking can fully activate the waist and abdomen, which has a significant effect on the improvement of waist and abdominal muscles [28].

Emotion can be said to be the external manifestation of a person's emotional state in a certain period of time, and emotional regulation is a process of effective regulation of the current emotional experience state in a purposeful and planned manner. Emotion regulation strategies are the internal mechanisms that guide how to effectively regulate emotions in this process. The use of positive and effective emotion regulation strategies can quickly improve a person's emotion, and in turn, a good emotion can also reflect a person's ability to regulate emotions better. In the process of individual emotion regulation, more active and effective emotion regulation strategies, such as cognitive reappraisal emotion regulation strategies, should be used.

*Collecting the Doctor's Diagnosis Data*. The doctor understands the condition through methods such as “look, smell, ask, and cut”, and after analyzing the condition through the examination data, he will make a diagnosis for the patient. However, there is also a process of change in the doctor's diagnosis, that is to say, the doctor's initial diagnosis of the patient (also referred to as the admission diagnosis) and the final diagnosis (also referred to as the “discharge diagnosis”) when the patient is cured (or transferred) may be different. At the same time, the same patient may be diagnosed with multiple diseases at the same visit, so it is possible to have multiple diagnoses. As the collection of medical big data, it is necessary to collect all the process data, which is one of the foundations of analysis. Every time a doctor diagnoses a patient, the diagnostic data are collected, not the final result [29].

For data acquisition, the higher the real-time performance, the closer the data is to the truth, and the higher the efficiency. However, for medical big data, the amount of data is very large, there are so many production links, the storage is also very scattered, and it also exists in heterogeneous information systems [30–32]. If the data are collected in real time, the transmission speed and stability of the network are highly required, and the existing hospital management information system will cause certain data pressure. After the doctor has diagnosed the patient's condition, he will issue a prescription for the treatment of the disease. The details of the prescription generally include drugs and treatment items. The data of drugs in the prescription details are as follows: drug name, usage and dosage, etc.; the data of treatment items: the name of treatment items, the frequency of treatment items, etc. It should be noted that the storage and management of the treatment items and the mentioned inspection items in the hospital's management information system (especially in the hospital management information system with charge management as the core) are the same. In the actual medical process, although the two have similarities, they are both medical items, and both are charged according to the item; but its fundamental purpose is different. General inspection items are mainly to provide data basis for diagnosis and have no therapeutic effect, while treatment items are mainly for the treatment of symptoms, and relatively few data items are involved. Therefore, when we collect inspection items and treatment items, we should pay attention to different treatment, and the data structure is also different [33]. The frequency of data collection needs to be carried out according to the characteristics of data and data use. In this study, the analysis of medical big data is mainly carried out. Using the analysis results to carry out intelligent supervision belongs to the auxiliary management system of big data applications, so the real-time requirements of the data are not strong. On the other hand, patient visits, doctor's diagnosis, prescription, etc. are generally performed only once a day. Therefore, when the system collects data, the commonly used data are collected once a day; the less commonly used data are collected once a week or a month. The collection time is set in the evening when there are almost no patients visiting a doctor, no medical staff operating the information system, and it is more suitable to collect data when the data is not updated [34, 35].

## 6. Conclusion

Emotion is a very important concept in psychology. Emotion is composed of multiple components, multiple dimension combinations, and multiple levels of integration. It is the psychological activity process and psychological motivation energy that interacts with cognition in the process of people's survival adaptation and interpersonal communication. Through the way of biofeedback, Taijiquan exercise can affect the individual's emotion, and Taijiquan exercise can promote the practitioner to maintain or improve the function of the nervous system, so that the individual's emotion is affected. In order to improve students' emotional management ability, this study tried to use Tai Chi combined with group work to intervene in the practice of students' emotional improvement. Its purpose is to help students learn the relevant knowledge of emotion management, reduce the trouble of negative emotions, and improve the ability of emotion regulation. Finally, the methods and skills in practice are summarized, which can provide reference for similar group work in the future. This study only confirms the effect of Taijiquan on the mental health of college students in physiological state but does not observe and evaluate the impact of Taijiquan on the mental health of college students in pathological state. It also needs to be supplemented by more work in the future to lay a solid theoretical foundation for the promotion of Taijiquan as an effective mental health intervention. Taijiquan practitioners should do a good job in organizing activities such as Taijiquan publicity and teaching on the basis of insisting on exercise and vigorously encourage and promote more people to participate in the ranks of Taijiquan training; furthermore, reading books related to Taijiquan exercise, on the basis of theoretical study, enhances the understanding of Taijiquan exercise concept and profound connotation and combines theory with practical activities, so as to better promote physical and mental health; college students who participate in other exercise methods can use their spare time to watch the Taijiquan exercise process, increase their interest in Taijiquan exercise, and actively participate in Taijiquan exercise, taking into account both the original physical exercise method and Taijiquan exercise. In addition to regulating emotions, Taijiquan should be used more for physical fitness in the future, and it should be promoted more.

## Figures and Tables

**Figure 1:** Logical structure of medical big data.

**Figure 2:** Network topology.

**Figure 3:** Before and after the third-grade experiment, the experimental class's and the control class's height and weight indicators compared with each other.

**Figure 4:** Changes in the average height and weight of fourth-grade students.

**Figure 5:** Comparison of 50  m running time between grades 3 and 4.

**Figure 6:** Students' physical fitness test results.

**Figure 7:** The state of mind of 12 people.

**Figure 8:** Intervention effect of group work on emotional intelligence level.

**Figure 9:** Statistical results of each dimension of the emotion state self-assessment.

**Table 1:** Taijiquan teaching progress.

Week	Teaching objectives	Time	During follow-up
1–2	Students initially master the origin of Taijiquan	25 min/day	2.16 ± 1.39
3	Learn the basic movements of Tai Chi	25 min/day	1.81 ± 1.21
4	Practice the whole set of moves independently	30 min/day	2.32 ± 1.44
5–14	Skilled practice	30 min/day	0.84 ± 0.73

**Table 2:** Comparison of different intervention time between Tai Chi training group and blank control group.

Different types	Different groups	Tai Chi training		Blank control	
		During the intervention	During follow-up	During the intervention	During follow-up
Low-intensity activities	1	1.85 ± 0.90	2.22 ± 1.33	1.73 ± 0.92	2.16 ± 1.39
	2	1.68 ± 0.65	1.67 ± 0.67	1.69 ± 0.61	1.81 ± 1.21
	3	1.94 ± 1.00	2.51 ± 1.49	1.75 ± 1.03	2.32 ± 1.44

Moderate-intensity activities	1	1.06 ± 0.33	0.85 ± 0.93	0.56 ± 0.37	0.84 ± 0.73
	2	1.10 ± 0.36	0.68 ± 0.79	0.56 ± 0.36	0.76 ± 0.79
	3	1.04 ± 0.32	0.94 ± 0.99	0.56 ± 0.38	0.88 ± 0.70

High-intensity activities	1	0.17 ± 0.22	0.22 ± 0.48	0.21 ± 0.32	0.23 ± 0.43
	2	0.29 ± 0.29	0.46 ± 0.73	0.45 ± 0.44	0.45 ± 0.65
	3	0.11 ± 0.14	0.09 ± 0.16	0.10 ± 0.16	0.13 ± 0.22

**Table 3:** GSES scoring results.

Gender type	Tai Chi training group (*n* = 95)		Blank control group (*n* = 103)	
	Before intervention	Intervention ends	Before intervention	Intervention ends
Gender neutral	2.55 ± 0.43	2.59 ± 0.43	2.47 ± 0.39	2.54 ± 0.44
Male	2.60 ± 0.48	2.63 ± 0.52	2.57 ± 0.35	2.65 ± 0.42
Female	2.53 ± 0.39	2.57 ± 0.37	2.42 ± 0.40	2.49 ± 0.44

**Table 4:** Comparison of SCL90 score results.

Gender type	Tai Chi training group (*n* = 95)		Blank control group (*n* = 103)	
	Before intervention	Intervention ends	Before intervention	Intervention ends
Gender neutral	162.84 ± 31.30	176.97 ± 31.47	168.27 ± 30.51	179.78 ± 32.50
Male	165.12 ± 35.58	173.69 ± 33.99	163.25 ± 29.68	129.21 ± 25.80
Female	161.62 ± 29.01	178.72 ± 30.18	150.53 ± 30.81	164.54 ± 34.22

**Table 5:** Comparison of height and weight of students in experimental class and control class.

Different factors	Third grade		Fourth grade	
	Height (cm)	Weight (kg)	Height (cm)	Weight (kg)

Experimental class (*x* ± *s*)	168.5 ± 6.86	46.01 ± 7.00	147.94 ± 5.04	56.8 ± 11.94
Control class (*x* ± *s*)	164.74 ± 7.25	50.94 ± 8.55	146.39 ± 3.65	54.3 ± 4.79
*F*	0.29	0.211	2.741	24.616
Sig	0.59	0.648	0.104	0.000
*T*	1.5	−0.38	1.266	0.974
Sig (both ± sides)	0.142 > 0.05	0.706 > 0.05	0.212 > 0.05	0.337 > 0.05

**Table 6:** Comparison of emotion factors.

Factor term	Control group	Tai Chi group
Activity	−0.15 ± 408	0.98 ± 2.75
Pleasure	0.19 ± 1.15	0.69 ± 2.35
Thoughtful	0.06 ± 1.02	0.19 ± 2.16
Calmness	0.16 ± 0.65	0.26 ± 2.34
Anger	−0.14 ± 1.14	−0.48 ± 1.79

## Data Availability

The data that support the findings of this study can be obtained from the corresponding author upon reasonable request.
